The article "Effects of the Wenyang Zhenshuai Granule on the Expression of LncRNA-MiR143HG/miR-143 Regulating ERK5 in H9C2 Cardiomyocytes" was retracted in 2023. Reasons: signs of a paper mill; compromised peer review; unreliable results or conclusions.

# Effects of the Wenyang Zhenshuai Granule on the Expression of LncRNA-MiR143HG/miR-143 Regulating ERK5 in H9C2 Cardiomyocytes

**DOI:** 10.1155/2021/6431007

**Published:** 2021-08-07

**Authors:** Zelin Xu, Xinyu Chen, Qingyang Chen, Huzhi Cai

**Affiliations:** The First Hospital of Hunan University of Chinese Medicine, Changsha 410007, Hunan, China

## Abstract

Chronic heart failure (CHF) is a complex clinical syndrome caused by a variety of heart problems, with a high incidence. The 5-year survival rate of patients with clinical symptoms is similar to that of malignant tumors. Wenyang Zhenshuai granules are a safe and effective granule of traditional Chinese medicine components, including aconite, dried ginger, licorice, and red ginseng. In contemporary clinical applications, it is widely used in acute and chronic heart insufficiency, coronary heart disease, and arrhythmia. This research cultured H9C2 cardiomyocytes and divided them into the normal control group, LncRNA-MiR143HG overexpression group, LncRNA-MiR143HG silence group, Adriamycin (ADR) group, ADR + medicated serum group, ADR + LncRNA-MiR143HG overexpression + medicated serogroup, and ADR + LncRNA-MiR143HG silence + medicated serogroup. The cells of each group were treated differently, and the survival rate of each group of cells and the expression levels of LncRNA-MiR143HG/miR-143 and ERK5 were detected at the end of the experiment, and the expression of LncRNA-MiR143HG/miR-143 in H9C2 cardiomyocytes was regulated by Wenyang Zhenshuai granules' impact. The results of this study showed that, in the doxorubicin-induced H9C2 cardiomyocyte injury model, the expression of miR-143 was upregulated, and the expression of LncRNA-MiR143HG and ERK5 was significantly downregulated. Wenyang Zhenshuai granules can downregulate the expression of miR-143 to promote ERK5 protein expression and phosphorylation. The process is regulated by LncRNA-MiR143HG/miR-143, which may be one of its important mechanisms for the treatment of chronic heart failure.

## 1. Introduction

Chronic heart failure (CHF) is a complex clinical syndrome caused by the progression of various heart diseases to severe stages. Its incidence is high. The 5-year survival rate of patients with clinical symptoms is similar to that of malignant tumors [1–3]. The previous research of the research group confirmed that the phosphorylation expression of ERK5 pathway protein, the main subfamily of mitogen-activated protein kinase (MAPK) signaling pathway, is closely and negatively correlated with the progression of CHF [4], and Wenyang Zhenshuai Granules can significantly upregulate the expression of ERK5 protein phosphorylation. Bioinformatics analysis shows that the 3′UTR of human ERK5 gene contains a putative consensus site (nucleotides 2917–2932) bound by microRNA-143 (miRNA-143) [5], and it is based on the luciferase reporter gene vector. The experiment verified the specificity of miR-143 and ERK5 in sequence binding and confirmed that there is a theoretical basis for interaction [6–8]. As the host gene of miR-143, long noncoding RNA-MiR143HG (lncRNA-MiR143HG) has been proven to directly regulate miR-143, and the regulation between the two plays an important role in the process of heart development and structure formation [9]. Through further research, we found that the specific role of the lncRNA-MiR143HG/miR-143/ERK5 regulatory system in the occurrence and development of chronic heart failure is still unclear. Whether Wenyang Zhenshuai granules regulates LncRNA-MiR143HG/miR-143. In turn, it affects the ERK5-mediated cardiomyocyte damage effect and produces a therapeutic effect. In order to answer this scientific question, we designed and completed this experiment.

The article "Effects of the Wenyang Zhenshuai Granule on the Expression of LncRNA-MiR143HG/miR-143 Regulating ERK5 in H9C2 Cardiomyocytes" was retracted in 2023. Reasons: signs of a paper mill; compromised peer review; unreliable results or conclusions.

## 2. Materials and Methods

### 2.1. Drugs and Reagents

Adriamycin hydrochloride was provided by Shenzhen Wanle Pharmaceutical Co., Ltd. (H44024359), SYBR Green PCR kit was purchased from Shanghai Sixin Biotechnology Co., Ltd. (BL705A), and Wenyang Zhenshuai granules were purchased from the First Affiliated Hospital of Hunan University of Traditional Chinese Medicine Provided (201902), and ERK5 and p-ERK5 antibodies were purchased from Wuhan Boster Bioengineering Co., Ltd. (ab40908, ab5686). LncRNA-MiR143HG overexpression and siRNA vector were purchased from Shanghai Ebers Biotechnology Co., Ltd.

### 2.2. Subculture of Cardiomyocyte Cell Lines

H9C2 cardiomyocytes (Shanghai Gefan Biological Cell Bank) were used, and the cells were passaged in DMEM medium with 10% FBS. When the cells became full at the bottom of the culture flask, 0.25% trypsin was added and the adherent cells were gently pipetted to make a single cell solution; the remaining cell suspension was diluted and then the cell count was performed, and the cell concentration was adjusted according to the counting result and planted in a plate for culture.

### 2.3. Preparation of Medicated Serum

We used distilled water to make 6 ml solution of Wenyang Zhenshuai granules (1.44 g/kg·d) into rats [4], gavage twice a day, 3 ml each time for 7 days; 7 days later, blood was taken from the abdominal aorta. The blood was centrifuged at 3000 r/min, the supernatant was taken, and the bacteria were removed by suction filtration, then aliquoted, stored in a refrigerator at −20°C for later use, and configured to be used at a concentration of 10% for experiments.

### 2.4. Transfection of LncRNA-MiR143HG Overexpression and Silence in Cardiomyocytes

1 × 10^5^ cells were seeded in a 6-well plate, and 10% FBS-containing medium was added to the culture. When the cell density reached 50%, the transfection was started. LncRNA-MiR143HG overexpression and siRNA vector were diluted with pure DMEM, mixed, and incubated at room temperature for 5 minutes to prepare a DNA and siRNA dilution. Lipo2000 was diluted in the corresponding amount of DMEM, allowed to stand for 5 minutes at room temperature, and incubated for 20 minutes at room temperature to form a transfection complex. The corresponding amount of the transfection complex was placed in an incubator and the medium was changed after 6 hours. After the culture was over, the expression of LncRNA-MiR143HG in cardiomyocytes after transfection was detected by RT-PCR to determine whether the overexpression and silent transfection were successful.

The article "Effects of the Wenyang Zhenshuai Granule on the Expression of LncRNA-MiR143HG/miR-143 Regulating ERK5 in H9C2 Cardiomyocytes" was retracted in 2023. Reasons: signs of a paper mill; compromised peer review; unreliable results or conclusions.

### 2.5. Induction of Cardiomyocyte Damage and Grouping

Adriamycin (ADR) was added to the cardiomyocyte culture medium of the ADR group, and the concentration was adjusted to 2.67 *μ*mol/L and cultured for 44 hours [10]. The cardiomyocytes were seeded in 6-well plates, and a total of 7 plates were seeded. Cells of each plate were grouped; they were divided into 7 groups, namely, the normal control group, LncRNA-MiR143HG overexpression group, LncRNA-MiR143HG silence group, ADR group, ADR + medicated serum group, ADR + LncRNA-MiR143HG overexpression + medicated serogroup, and ADR + LncRNA-MiR143HG silence + medicated serogroup.

### 2.6. Morphological Observation and Survival Rate Detection of Cardiomyocytes

After the experiment, the cardiomyocytes of each group were taken, and the morphological changes of the cardiomyocytes of each group were observed with an inverted microscope. After the experiment was completed, the cardiomyocytes of each group were collected, the cell suspension concentration was adjusted, 20 *μ*l/ml MTT solution was added to the medium, the cell supernatant after MTT culture was sucked, DMSO solution was added, and the culture plate was shaken on a shaker at low speed for 10 minutes, and the absorbance value of each group of cells was detected by enzyme-linked immunosorbent assay at 490 nm. The greater the absorbance value, the higher the survival rate.

### 2.7. Detection of LncRNA-MiR143HG, miR-143, and ERK5 Gene Expression in Cardiomyocytes

The cardiomyocytes of each group were taken out, and primers were designed according to the LncRNA-MiR143HG, miR-143, and ERK5 gene sequences in the NCBI gene bank. The total RNA was extracted by Trizol in one step and stored at −80°C. Fluorescence quantitative RT-PCR analysis of LncRNA-MiR143HG, miR-143, and ERK5 was performed in accordance with the PCR reaction kit instructions, and 2^−ΔΔCt^ was used to calculate the multiple relationship between the target gene expression of the experimental group and the control group: △△CT = △CT_experimental group_−△CT_control group_; △CT_experimental group_ = CT_target gene, experimental group_ − CT_internal reference gene, experimental group_; △CT_control group_ = CT_target gene, control group_ − CT_internal reference gene, control group_. The primer design is shown in Table 1.

The article "Effects of the Wenyang Zhenshuai Granule on the Expression of LncRNA-MiR143HG/miR-143 Regulating ERK5 in H9C2 Cardiomyocytes" was retracted in 2023. Reasons: signs of a paper mill; compromised peer review; unreliable results or conclusions.

### 2.8. Detection of ERK5 and p-ERK5 Protein Expression in Cardiomyocytes

SDS buffer was added to 50 *μ*g of total cardiomyocyte protein, and the cells were denatured at 100°C for 8 minutes with a constant current. The first 15 minutes were electrophoresed at 16 mA/gel, and then 32 mA/gel was electrophoresed to the bottom. The electroswitching mode set the current according to the film area of 0.8 mA/cm2, and the film was transferred for 2 h. ERK5 (1 : 1000) total protein and p-ERK5 (1 : 1000) protein primary antibodies were added separately and kept at 4°C overnight. Enzyme-labeled secondary antibody was added and hybridized at room temperature for 2 hours. TBST was rinsed for 10 min × 3 times. ECL was used for exposure, followed by visualization, scanning, saving, and analysis.

### 2.9. Statistics Methods

All data were tested for normality and processed with SPSS17.0 statistical analysis software package. Measurement data were all expressed. Single-factor analysis of variance was used for comparison between groups of averages and groups. LSD method was used for homogeneous variances, and Tamhane's T2 method was used for uneven variances. *P* < 0.05 indicates statistical difference.

## 3. Results

### 3.1. Morphological Observation of Myocardial Cells in Each Group

Under an inverted microscope, cardiomyocytes in the normal control group, LncRNA-MiR143HG overexpression group, and LncRNA-MiR143HG silence group were arranged neatly, in a regular spindle or polygonal shape, with a sense of three-dimensionality and refraction; in the ADR group, there were wrinkles shrinkage, cells appeared flat, gaps became larger, and volume became smaller. The degeneration of cardiomyocytes in the ADR + medicated serum group, ADR + LncRNA-MiR143HG overexpression + medicated serogroup, and ADR + LncRNA-MiR143HG silence + medicated serogroup was improved compared with the ADR group. Among them is ADR + LncRNA, The improvement of MiR143HG overexpression + medicated serogroup was the most obvious as shown in Figure 1.

### 3.2. Comparison of the Survival Rate of Cardiomyocytes in Each Group

After the experiment, the comparison of the survival rate of cardiomyocytes in each group showed that the survival rate of the normal control group, the LncRNA-MiR143HG overexpression group, and the LncRNA-MiR143HG silence group were similar, and the difference was not statistically significant (*P* > 0.05). Compared with the normal control group, the cell survival rate of ADR group, ADR + medicated serum group, ADR + LncRNA-MiR143HG overexpression + medicated serogroup, and ADR + LncRNA-MiR143HG silence + medicated serogroup was significantly decreased compared with the normal control group. The difference was statistically significant (*P* < 0.05). ADR + medicated serogroup, ADR + LncRNA-MiR143HG overexpression + medicated serogroup, ADR + LncRNA-MiR143HG silence + medicated serogroup compared with ADR group, and the cell survival rate increased; the difference was statistically significant (*P* < 0.05). The ADR + medicated serum group and ADR + LncRNA-MiR143HG overexpression + medicated serogroup had a higher cell survival rate than the ADR + LncRNA-MiR143HG silence + medicated serogroup, and the difference was statistically significant (*P* < 0.05) as shown in Figure 2.

The article "Effects of the Wenyang Zhenshuai Granule on the Expression of LncRNA-MiR143HG/miR-143 Regulating ERK5 in H9C2 Cardiomyocytes" was retracted in 2023. Reasons: signs of a paper mill; compromised peer review; unreliable results or conclusions.

### 3.3. Expression of LncRNA-MiR143HG, miR-143, and ERK5 Genes in Cardiomyocytes of Each Group

After the experiment, the expression of LncRNA-MiR143HG in myocardial cells of each group was compared. The expression of LncRNA-MiR143HG in the LncRNA-MiR143HG overexpression group was significantly higher than that in the normal control group. The expression of LncRNA-MiR143HG in the LncRNA-MiR143HG silence group was significantly lower than that of the normal control group, and the difference was statistically significant (*P* < 0.05). Compared with the normal control group, the expression of LncRNA-MiR143HG in ADR group, ADR + medicated serum group, ADR + LncRNA-MiR143HG overexpression + medicated serogroup, and ADR + LncRNA-MiR143HG silence + medicated serogroup was significantly decreased. The difference is statistically significant (*P* < 0.05). Compared with the ADR group and ADR + LncRNA-MiR143HG silence + medicated serogroup, the expression of LncRNA-MiR143HG in the ADR + medicated serum group, ADR + LncRNA-MiR143HG overexpression + medicated serogroup increased, and the difference was statistically significant (*P* < 0.05). The expression of LncRNA-MiR143HG decreased in the ADR + LncRNA-MiR143HG silence + medicated serogroup compared with the ADR group, and the difference was statistically significant (*P* < 0.05) as shown in Figure 3.

After the experiment, the expressions of miR-143 genes in cardiomyocytes of each group were compared. The expressions of miR-143 in the normal control group, LncRNA-MiR143HG overexpression group, and LncRNA-MiR143HG silence group were similar, and the difference was not statistically significant (*P* > 0.05). The ADR group, ADR + medicated serum group, ADR + LncRNA-MiR143HG overexpression + medicated serogroup, and ADR + LncRNA-MiR143HG silence + medicated serogroup were compared with the normal control group, and the expression of miR-143 in cells was obviously rising; the difference was statistically significant (*P* < 0.05). Compared with the ADR group and the ADR + LncRNA-MiR143HG silence + medicated serogroup, the ADR + medicated serum group and ADR + LncRNA-MiR143HG overexpression + medicated serogroup showed a decrease in the expression of miR-143. Compared with the ADR group, the expression of miR-143 in the +LncRNA-MiR143HG silence + medicated serogroup was significantly increased, and the difference was statistically significant (*P* < 0.05) as shown in Figure 4.

The article "Effects of the Wenyang Zhenshuai Granule on the Expression of LncRNA-MiR143HG/miR-143 Regulating ERK5 in H9C2 Cardiomyocytes" was retracted in 2023. Reasons: signs of a paper mill; compromised peer review; unreliable results or conclusions.

After the experiment, the expressions of ERK5 genes in cardiomyocytes of each group were compared. The expressions of ERK5 in the normal control group, LncRNA-MiR143HG overexpression group, and LncRNA-MiR143HG silence group were similar, and the difference was not statistically significant (*P* > 0.05). The ADR group, ADR + medicated serum group, ADR + LncRNA-MiR143HG overexpression + medicated serogroup, and ADR + LncRNA-MiR143HG silence + medicated serogroup were compared with the normal control group; the cell ERK5 expression was significantly decreased. The differences are all statistically significant (*P* < 0.05). The ADR + medicated serum group and ADR + LncRNA-MiR143HG overexpression + medicated serogroup had increased cell ERK5 expression compared with the ADR group, and the difference was statistically significant (*P* < 0.05). Compared with the ADR + LncRNA-MiR143HG silence + medicated serogroup, the ADR + medicated serum group, and ADR + LncRNA-MiR143HG overexpression + medicated serogroup had higher cell ERK5 expression, and the difference was statistically significant (*P* < 0.05). There was no significant difference between the ADR + LncRNA-MiR143HG silence + medicated serogroup and the ADR group (*P* > 0.05) as shown in Figure 5.

### 3.4. Expression of p-ERK5 and ERK5 in Cardiomyocytes of Each Group

After the experiment, the expression of p-ERK5 and ERK5 in cardiomyocytes of each group showed that the expression of P-ERK5 and ERK5 protein in the normal control group, LncRNA-MiR143HG overexpression group, and LncRNA-MiR143HG silence group were equivalent, and the difference was not statistically significant (*P* > 0.05). Compared with the normal control group, ADR group, ADR + medicated serum group, and ADR + LncRNA-MiR143HG silence + medicated serogroup, the expression of P-ERK5 and ERK5 protein in cells decreased significantly, and the difference was statistically significant (*P* < 0.05). ADR + medicated serum group, ADR + LncRNA-MiR143HG overexpression + medicated serogroup, and ADR + LncRNA-MiR143HG silence + medicated serogroup were compared with ADR group; the expression of P-ERK5 and ERK5 protein in cells had risen, and the difference was statistically significant (*P* < 0.05). Compared with the ADR + LncRNA-MiR143HG silence + medicated serogroup, the ADR + medicated serum group and ADR + LncRNA-MiR143HG overexpression + medicated serogroup had higher cell P-ERK5 protein expression, and the difference was statistically significant (*P* < 0.05). The ADR + LncRNA-MiR143HG overexpression + medicated serogroup had higher cell ERK5 protein expression than the ADR + LncRNA-MiR143HG silence + medicated serogroup, and the difference was statistically significant (*P* < 0.05); ADR + LncRNA-MiR143HG overexpression + medicated serogroup was compared with normal control group, and ERK5 protein expression was not statistically different (*P* > 0.05) as shown in Figure 6.

The article "Effects of the Wenyang Zhenshuai Granule on the Expression of LncRNA-MiR143HG/miR-143 Regulating ERK5 in H9C2 Cardiomyocytes" was retracted in 2023. Reasons: signs of a paper mill; compromised peer review; unreliable results or conclusions.

## 4. Discussion

Cells are the basic structures that make up life, and changes in cell structure and function are based on a series of intracellular signal transduction. ERK5 is an atypical pathway in the MAPK family. It is mainly located in the cytoplasm. It receives signals from outside the cell and is activated by its upstream kinase MEK5. It can then be transferred to the nucleus to phosphorylate the transcription factor cardiomyocyte enhancer and regulate its transcription active [11, 12]. Since ERK5 was cloned for the first time by Zhou et al. [13] in 1995, it has been found to control a series of functions originally thought to be completed by ERK1/2, and it is clear that it is in oxidative stress, hypoxia, reactive oxygen species, and various mitoses. Under the original excitement, it plays an important role in maintaining the integrity of blood vessels and the development of the heart. A large number of documents have shown that the medicines of traditional Chinese medicine have good effects on treating heart failure and other diseases [14, 15]. Wenyang Zhenshuai granules contain a variety of Chinese herbal medicine ingredients. From the previous research results of the research group, Wenyang Zhenshuai granules not only can activate p-ERK5 but also have obvious and beneficial regulatory effects on the main downstream active components MEF-2 and CREB through the ERK5 pathway. miR-143 is located in the long arm of human chromosome 5, zone 3, and zone 2. Its function mainly affects the expression of related specific proteins by regulating the posttranscriptional level and inhibiting the translation of target genes. Through bioinformatics analysis and luciferase reporter gene vector experiment verification, it is presumed that the direct target gene of miR-143 is ERK5 [16]. Zheng [7] et al. proved that upregulation of miR-143 can significantly reduce the expression of p-ERK5 and ERK5 in cells, while downregulation of miR-143 has the opposite effect. As the host gene of miR-143, lncRNA-MiR143HG can directly regulate miR-143 and thus affect the development and function of the heart [9], and studies have shown that lncRNA-MiR143HG is significantly upregulated during myocardial remodeling in patients with aortic stenosis. It is suggested that it is involved in the process of myocardial remodeling [17]. In view of the abovementioned preliminary research results, LncRNA-MiR143HG regulates miR-143 and affects the signal pathway of ERK5, which is of great research value.

The article "Effects of the Wenyang Zhenshuai Granule on the Expression of LncRNA-MiR143HG/miR-143 Regulating ERK5 in H9C2 Cardiomyocytes" was retracted in 2023. Reasons: signs of a paper mill; compromised peer review; unreliable results or conclusions.

Wenyang Zhenshuai ganules is an in-hospital preparation of the First Affiliated Hospital of Hunan University of Traditional Chinese Medicine presided over by Professor Chen Xinyu. Before being developed into granules, its basic decoction has been safely and effectively used in the First Affiliated Hospital of Hunan University of Traditional Chinese Medicine for nearly ten years. Its prescription includes aconite, dried ginger, licorice, and red ginseng. Aconite warms the kidney and yang, and dried ginger nourishes the spleen yang, and the two go one by one, help the yang, break the yin, and save the adversity by eliminating the cold [18, 19]. Licorice is used to regulate and invigorate deficiency [20]. In contemporary clinical applications, it is not only widely used in acute and chronic cardiac insufficiency, coronary heart disease, arrhythmia, and so on but also used for warming yang and qi to treat cardiogenic or renal origin, edema. On the basis of Sini Decoction, red ginseng is added to warm the yang to invigorate the qi, restore the pulse, and relieve the blood, which not only has the effect of regaining the yang and relieving adversity but also has the ability to warm the meridians and collaterals.

The previous research of the research group found that Wenyang Zhenshuai granules can effectively improve the symptoms of chronic heart failure induced by Adriamycin in experimental animals and can significantly increase the expression of myocardial ERK5 protein phosphorylation. This experimental study found that in normal H9C2 cells, after overexpression and silencing of LncRNA-MiR143HG, the cell morphology, survival rate, miR-143, and ERK5 expression did not change significantly, but in the case of H9C2 cardiomyocyte damage induced by doxorubicin in the model, the cell morphology was malignant, the survival rate was reduced, the expression of LncRNA-MiR143HG and ERK5 decreased significantly, and the expression of miR-143 increased significantly. The cell morphology of the group treated with Wenyang Zhenshuai granules gradually returned to normal, the survival rate was significantly increased, the expression of LncRNA-MiR143HG and ERK5 was significantly upregulated, and the expression of miR-143 was significantly reduced. After regulating LncRNA-MiR143HG, in the ADR model, the intervention of Wenyang Zhenshuai granules promoted the regulation of LncRNA-MiR143HG, which caused changes in the expression of miR-143, thereby causing changes in the expression of ERK5. The above experimental results indicate that the expression of LncRNA-MiR143HG and miR-143 plays an important regulatory role in the process of cardiomyocyte injury and is closely related to the expression of ERK5. Wenyang Zhenshuai granules may regulate LncRNA-MiR-143 in H9C2 cardiomyocytes. The expression of MiR143HG and miR-143 in turn affects the cardiomyocyte protection mediated by ERK5.

The article "Effects of the Wenyang Zhenshuai Granule on the Expression of LncRNA-MiR143HG/miR-143 Regulating ERK5 in H9C2 Cardiomyocytes" was retracted in 2023. Reasons: signs of a paper mill; compromised peer review; unreliable results or conclusions.

## 5. Conclusion

In summary, Wenyang Zhenshuai granules can downregulate the expression of miR-143 to promote ERK5 protein expression and phosphorylation, and the related process is regulated by LncRNA-MiR143HG/miR-143, which may be one of its important mechanisms for the treatment of chronic heart failure. But the specific control process still needs in-depth study.

## Figures and Tables

**Figure 1:** Morphological observation of cardiomyocytes in each group after the experiment (×100). (a) Normal control group, (b) LncRNA-MiR143HG overexpression group, (c) LncRNA-MiR143HG silence group, (d) ADR group, (e) ADR + medicated serum group, (f) ADR + LncRNA-MiR143HG overexpression + medicated serogroup, and (g) ADR + LncRNA-MiR143HG silence + medicated serogroup.

**Figure 2:** Comparison of the survival rate of cardiomyocytes in each group. Note: compared with the normal control group, ^*∗*^*P* < 0.05; compared with the ADR group, ^#^*P* < 0.05; compared with the ADR + LncRNA-MiR143HG silence + medicated serogroup, ^+^*P* < 0.05.

**Figure 3:** Comparison of LncRNA-MiR143HG expression in cardiomyocytes of various groups. Note: compared with the normal control group, ^*∗*^*P* < 0.05; compared with the ADR group, ^#^*P* < 0.05; compared with the ADR + LncRNA-MiR143HG silence + medicated serogroup, ^+^*P* < 0.05.

**Figure 4:** Comparison of miR-143 expression in cardiomyocytes of various groups. Note: compared with the normal control group, ^*∗*^*P* < 0.05; compared with the ADR group, ^#^*P* < 0.05; compared with the ADR + LncRNA-MiR143HG silence + medicated serogroup, ^+^*P* < 0.05.

The article "Effects of the Wenyang Zhenshuai Granule on the Expression of LncRNA-MiR143HG/miR-143 Regulating ERK5 in H9C2 Cardiomyocytes" was retracted in 2023. Reasons: signs of a paper mill; compromised peer review; unreliable results or conclusions.

**Figure 5:** Comparison of ERK5 expression in cardiomyocytes of various groups. Note: compared with the normal control group, ^*∗*^*P* < 0.05; compared with the ADR group, ^#^*P* < 0.05; compared with the ADR + LncRNA-MiR143HG silence + medicated serogroup, ^+^*P* < 0.05.

**Figure 6:** Comparison of the expression of p-ERK5 and ERK5 proteins in cardiomyocytes of each group. (a) Normal control group, (b) LncRNA-MiR143HG overexpression group, (c) LncRNA-MiR143HG silence group, (d) ADR group, (e) ADR + medicated serum group, (f) ADR + LncRNA-MiR143HG overexpression + medicated serogroup, and (g) ADR + LncRNA-MiR143HG silence + medicated serogroup. Compared with the normal control group, ^*∗*^*P* < 0.05; compared with the ADR group, ^#^*P* < 0.05; compared with the ADR + LncRNA-MiR143HG silence + medicated serogroup, ^+^*P* < 0.05.

**Table 1:** qRT-PCR primers.

Primer sequence	Forward (5′-3′)	Reverse (5′-3′)
LncRNA-MiR143HG	CAGCTCCCAGAACTCGTCCC	CCTCGTCTCCTTTTCCCATGTCT
miR-143	CGCCTGAGATGAAGCACTGTAG	CCAGGAGAAGGGGTGTTAGA
ERK5	CAATGCCAAACGGACCCTC	CTGAATTCTCCATAGGGCACAAT
5S	GCCTACAGCCATACCACCCGGAA	CCTACAGCACCCGGTATCCCA
GAPDH	ACAGCAACAGGGTGGTGGAC	TTTGAGGGTGCAGCGAACTT

## Data Availability

The datasets used and/or analyzed during the current study are available from the corresponding author upon reasonable request.
